# Potassium Channel Ether à go-go1 Is Aberrantly Expressed in Human Liposarcoma and Promotes Tumorigenesis

This article has been retracted.

**DOI:** 10.1155/2014/345678

**Published:** 2014-07-20

**Authors:** Jin Wu, Daixing Zhong, Yujian Wei, Xinyu Wu, Liangqi Kang, Zhenqi Ding

**Affiliations:** ^1^Department of Orthopaedics, the Affiliated Southeast Hospital of Xiamen University, Orthopaedic Center of People's Liberation Army, Zhanghua Road 269, Zhangzhou 363000, China; ^2^Department of Thoracic Surgery, the Affiliated Tangdu Hospital of Fourth Military Medical University, Xi'an 710038, China; ^3^School of Basic Medical College, Nanjing Medical University, Nanjing 210000, China; ^4^Department of Neurology, the Affiliated Southeast Hospital of Xiamen University, Zhangzhou 363000, China

## Abstract

The ether à go-go1 (Eag1) channel is overexpressed in a variety of cancers. However, the expression and function of Eag1 in liposarcoma are poorly understood. In the present study, the mRNA expression of Eag1 in different adipose tissue samples was examined by real-time PCR. Then, the protein expression of Eag1 in 131 different adipose tissues from 109 patients was detected by immunohistochemistry. Next, the associations between Eag1 expression and clinicopathological features of liposarcoma were analyzed. In addition, the effects of Eag1 on liposarcoma cell proliferation and cycle were evaluated by CCK-8, colony formation, xenograft mouse model, and flow cytometry, respectively. Finally, the activation of p38 mitogen-activated protein kinase (MAPK) was detected by Western blot analysis to explain the detailed mechanisms of oncogenic potential of Eag1 in liposarcoma. It was found that Eag1 was aberrantly expressed in over 67% liposarcomas, with a higher frequency than in lipoma, hyperplasia, inflammation, and normal adipose tissues. However, Eag1 expression was not correlated with clinicopathological features of liposarcoma. Eag1 inhibitor imipramine or Eag1-shRNA significantly suppressed the proliferation of liposarcoma cells *in vitro* and *in vivo*, accompanying with accumulation of cells in the G1 phase. These results suggest that Eag1 plays an important role in regulating the proliferation and cell cycle of liposarcoma cells and might be a potential therapeutic target for liposarcoma.

## 1. Introduction

Liposarcoma is a malignant tumor that arises in fat cells, first described by Virchow [1]. Liposarcoma is the most common soft tissue sarcoma in adults with the peak prevalence between 40 and 60 years of age and accounts for up to 20% of all soft tissue sarcomas [2, 3]. Liposarcoma occurs in almost any part of the body, mainly in the trunk, the limbs, and the abdominal cavity. Usually, lumps with painless and slow growing are the initial symptoms. Unfortunately, tumors in the abdomen can grow to be quite large before they are found. Soft tissue liposarcomas have been categorized into four distinct histological subtypes: well differentiated, myxoid, pleomorphic, and round cell [2, 4]. While well differentiated tumors have a favorable outcome with a 5-year survival rate of 75–100%, round cell and pleomorphic liposarcomas have the worst prognosis with 0–20% survival rate at 5 years [5].

In recent years, the functional role of voltage-gated K^+^ channels (Kv channels) in tumorigenesis has been an area of intense investigation [6]. Several Kv channels, especially Eag1 (Kv10.1,* KCNH1*) channels, are crucially implicated in tumor growth, progression, and metastasis [7–9]. Eag1 is a central nervous system- (CNS-) localized channel that is found ectopically expressed in several tumors [10, 11]. In addition, suppression of Eag1 expression in several cancer cell lines causes a significant reduction of cell proliferation, while ectopic expression of Eag1 induces aggressive tumors in immune deficient mice [12–14]. Collectively, these data support the oncogenic potential of Eag1 [13, 15]. However, up to now only one study has examined the expression of Eag1 in liposarcoma but did not investigate the role of Eag1 in detail [16]. Therefore, in this study, we first detect the expression of Eag1 in different adipose tissues diseases and analyze the association between Eag1 expression and clinicopathological features of liposarcoma. Next we examined the effects of an Eag1 inhibitor or Eag1 siRNA on liposarcoma cell proliferation, colony formation, tumor growth, and cell cycle* in vitro* and* in vivo*. Finally, we investigated signaling mechanism by which Eag1 promotes liposarcoma cell growth and cycle.

## 2. Materials and Methods

### 2.1. Sample Collection

A total of 131 formalin-fixed, paraffin-embedded specimens, including 80 liposarcomas from 65 patients, 19 lipomas from 17 patients, 15 hyperplasia of adipose tissues from 10 patients, 8 panniculitis from 8 patients, and 9 normal adipose tissues from 9 patients, were acquired from the affiliated Southeast Hospital of Xiamen University between January 2010 and June 2013, with complete clinicopathologic parameters. Confirmed healthy human brain obtained from biopsy and skeletal muscle from patients who underwent orthopedic surgery were used as a positive and negative control, respectively [14, 16]. All the specimens were obtained after obtaining written informed consent according to a protocol approved by the Institutional Review Board of the affiliated Southeast Hospital of Xiamen University.

### 2.2. PCR

Genomic DNA and total RNA were extracted using TRIzol reagent (Invitrogen, Rockville, MD, USA) according to the manufacturer's protocol. Two micrograms of RNA were subjected to reverse transcription. Sequences of forward and reverse primers, amplified fragment sizes, and annealing temperatures were as follows: Eag1, 5′-GCT TTT GAG AAC GTG GAT GAG-3′, 5′-CGA AGA TGG TGG CAT AGA GAA-3′, 475 bp, 56°C. glyceraldehyde-3-phosphate dehydrogenase (GAPDH), 5′-GCC TCA AGA TCA GCA AT-3′, 5′-AGG TCC ACC ACT GAC ACG TT-3′, 310 bp, 56°C. Quantitative RT-PCR was performed using an ABI Prism 7,000 sequence detector (Applied Biosystems) and the results were analyzed by the relative standard curve method (User Bulletin #2 of ABI Prism 7,700 Sequence Detection Systems, Applied Biosystems).

### 2.3. Immunohistochemical Staining

The tissue slide was baked in a dry oven at 60°C for 2 h to remove the coated paraffin. The samples were demineralized with an equal parts mixture of 20% sodium citrate and 45% formic acid. The slide was immersed twice in xylene for 3 min, hydrated with 100%, 95%, 70%, and 50% ethanol, and rinsed with cold tap water for 5 min. After dewaxing and blocking endogenous peroxidases, the sections were treated at 100°C in EDTA (1 mM, pH 8.0) for antigen retrieval and then incubated with Eag1 polyclonal antibody (ab86204, Abcam, Cambridge, MA, 1 : 300) overnight at 4°C. The slides were washed with PBS and incubated with horseradish peroxidase conjugated goat anti-rabbit IgG at room temperature for 1 h. Diaminobenzidine (DAB, Zhongshan Biotechnology, Beijing, China) was used to visualize the tissue slide and the sections were counterstained with haematoxylin. Samples were defined as positive when more than 10% of the cells stained positive with Eag1 antibody. Eag1 staining was classified as 0 (less than 10% of the tumor cells show staining), 1+ (faint staining in more than 10% of the cells), 2+ (moderate staining in more than 10% tumor cells), and 3+ (strong staining in more than 10% of the cells) and the immunohistochemical score was evaluated as negative (0), positive (1), and strongly positive (2 and 3) as described previously [17].

### 2.4. Cell Culture and Drugs

Human liposarcoma cell line SW-872 (HTB-92), 93T449 (CRL-3043), and human embryonic kidney cell line 293 (HEK293) were purchased from the American Type Culture Collection (ATCC, Rockville, MD, USA). SW-872 cells were cultured in MEM (minimum essential medium) media (Gibco, Rockville, MD, USA), supplemented with 10% (v/v) fetal bovine serum (FBS) (Gibco), 100 IU/mL penicillin, and 100 *μ*g/mL streptomycin in a humidified atmosphere of 5% CO_2_ at 37°C. 93T449 and HEK293 cells were cultured in RPMI-1640 medium (Gibco), supplemented with 10% FBS, 100 U/mL penicillin, and 100 *μ*g/mL streptomycin in a humidified atmosphere of 5% CO_2_ at 37°C. All cells were subcultured every 3-4 days. Imipramine was purchased from Sigma (St. Louis, MO, USA), dissolved in distilled water as 1 mM stock solution and stored at −20°C.

### 2.5. Preparation of Adenoviral shRNA Vectors

The oligonucleotides targeting human Eag1 were designed and selected as the template: AGC CAT CTT GGT CCC TTA TAA, which shared no homology with other coding sequences in human by BLAST analysis. A ring sequence of 9 base pairs (TTC AAG ACG) existed between the sense and antisense strands. The shRNA was synthesised by Sangon Biotech (Shanghai, China). Plasmid pGeneSil-1 was purchased from GeneSil Biotechnology (Wuhan, China), which contained the human U6 promoter inserted between BamHI and HindIII sites. The shRNA cassette was subcloned into pAdTrack vector between HindIII and XbaI sites. The recombinant plasmid was linearized by digestion with restriction endonuclease and subsequently cotransformed into* E. coli* BJ5183 cells with an adenoviral backbone plasmid pAdEasy-1. Recombinant plasmids were selected for kanamycin resistance and transfected into HEK293 cells. A recombinant adenovirus expressing shRNA against Eag (Ad5-Eag1-shRNA) was generated. The recombinant adenovirus control (Ad5-Control-shRNA), which carried a sequence of CTA GGT GTT CTA GTC TGG ACT and did not target any known human genes, was generated as control. All viruses were propagated and purified on a CsCl gradient using standard methods. Functional titer (plaque forming units) was determined with a plaque assay on HEK293 cells according to the method developed by Quantum Biotechnology.

### 2.6. Adenovirus Infection

Human liposarcoma cells (1 × 10^5^) in serum-free media were infected with Ad5-Eag1-shRNA or Ad5-Control-shRNA at 5 MOI (multiplicity of infection, calculated as PFU/cell numbers) in a humidified atmosphere of 5% CO_2_ at 37°C. Virus containing medium was removed 8 h later and replaced with fresh MEM medium containing 10% (v/v) FBS. Cells were incubated for another 48 h.

### 2.7. Cell Proliferation Assay

Cell proliferation was analyzed by using Cell Counting Assay Kit-8 (CCK-8) (Dojindo Molecular Technologies, Gaithersburg, MD) according to the manufacturer's protocol. Briefly, 5 × 10^3^ cells were starved in serum-free medium for 12 h and then the cells were infected with vectors or exposed to 20 *μ*M imipramine. After 96 h, the cells were harvested. Ten microliters of CCK-8 solution was added to each well, the cells were incubated for 1 h, and the absorbance (A) at 490 nm was measured by using spectrophotometer (Bio-Rad, Richmond, CA). Experiments were performed at least three times with representative data presented.

### 2.8. Colony Formation Assay

For colony formation assay, cells were seeded at 300 per 60 mm dish in triplicate and cultured to 2 weeks. The assay was stopped when the colonies are clearly visible even without looking under the microscope. Cell colonies were fixed and stained with 0.25% crystal violet in 50% ethanol for 20 to 30 min and then air dried and counted. The colony formation ratio was calculated according to the following formula: colony formation ratio (%) = (colony number/seeded cell number) × 100%.

### 2.9. Tumorigenicity Assay in Nude Mice

Thymus-null BALB/c nude mice (female, 4–6 weeks old) were obtained from the Animal Center of Chinese Academy of Medical Sciences. All animal procedures were performed according to approved protocols and in accordance with recommendations for the proper use and care of laboratory animals. Liposarcoma xenografts were established in nude mice as described previously [18, 19]. The liposarcoma-bearing mice were randomly divided into 3 groups (*n* = 6). Group 1 received intratumor injection with Ad5-Eag1-shRNA (10 MOI) every 3 days (6 injections totally). Group 2 received intratumor injections of Ad5-Control-shRNA (10 MOI) every 3 days (6 injections totally). Group 3 received normal saline injection as controls. Tumor growth was measured using caliper, and tumor volume (mm^3^) was determined with formula *ab* ^2^/2, where *a* was the length and *b* was the width of the tumor.

### 2.10. Flow Cytometry Analysis

The cells were collected and washed twice with cold PBS following the infection with shRNA for 48 h, and then cell pellets were resuspended at 1 × 10^6^ cells/mL and fixed in 70% cold ethanol overnight at 4°C. A fluorochrome solution containing 50 *μ*g/mL PI, 3.4 mmol/L sodium citrate, 20 *μ*g/mL RNase A, and 1% Triton X-100 was added and the mixture was incubated in the dark at room temperature for 30 min. The distribution of the cell cycle was measured using flow cytometry (FCM; Partec, Münster, Germany). FCM analysis was performed using the Cell Quest software (Beckton Dickinson, Franklin Lakes, NJ, USA).

### 2.11. Western Blot Analysis

5-6 × 10^7^ cells were collected and lysed in ice-cold lysis buffer containing 50 mmol/L Tris-Cl (pH 7.5), 150 mmol/L NaCl, 0.2 mmol/L EDTA, 1 mmol/L PMSF, and 1% (v/v) Nonidet-P40 for 30 min. The lysates were centrifuged at 13,200 rpm for 10 min at 4°C and the supernatants were collected. 25 *μ*g proteins were resolved by a 12% SDS-PAGE and blotted on nitrocellulose membranes (Bio-Rad). Membranes were blocked with 10% (w/v) nonfat milk powder at room temperature for 1 h and then incubated with antibodies against Eag1 (Abcam), p38 MAPK, phospho-p38 MAPK, and GAPDH (Cell Signaling Technology, Danvers, MA) overnight at 4°C, followed by incubation with horseradish peroxidase-conjugated goat anti-rabbit or anti-mouse secondary antibody (Santa Cruz Biotechnology, CA, USA) for 1 h at room temperature. Finally, the membranes were developed with chemiluminescent detection kit (Zhongshan Biotechnology). Experiments were performed at least three times with representative data presented.

### 2.12. Statistical Analysis

All data were presented as mean ± standard deviation (SD). Statistical significance was determined using analysis of variance (ANOVA) or *χ* ^2^-test using the SPSS18.0 program. *P* < 0.05 was considered as significant difference.

## 3. Results

### 3.1. Eag1 Is Frequently Aberrantly Expressed in Human Liposarcoma Specimens

First, we compared the mRNA expression level of Eag1 in different adipose tissue samples by real-time PCR. There was a clear increase in Eag1 mRNA level in liposarcoma samples (*n* = 3), compared to other tissues (*n* = 3) (Figure 1(a)). Next, Eag1 polyclonal antibody was employed for immunohistochemical staining. Positive Eag1 staining was detected in 54/80 (67.5%) liposarcoma, 8/19 (42.1%) lipoma, 6/15 (40.0%) hyperplasia of adipose tissues, and 2/8 panniculitis (25.0%), but negative Eag1 staining was detected in 9 normal adipose tissues (Table 1). The positive signal was detected mainly in the cytoplasm, consistent with previous reports [11, 16]. As a positive control Eag1 staining was detected in a normal human brain sample, negative staining for Eag1 was observed in a skeletal muscle tissue. The representative images of Eag1 staining are shown in Figure 1(b). Statistical analysis indicated that positive expression of Eag1 in human liposarcoma was significantly different from that in other adipose tissues diseases (*P* < 0.05, Table 1).

### 3.2. Clinical Parameters of Liposarcoma Specimens and Eag1 Expression

The clinical parameters of 80 liposarcoma specimens are shown in Table 2. Thirty-three (41.2%) males and 47 (58.8%) females with mean age of 47.98 ± 14.56 years (range 7–79 years) were enrolled in this study. Twenty-one (26.2%) tumors originated in the limbs, 23 (28.8%) in the trunk, 21 (26.2%) in the abdominal cavity, and 15 (18.8%) in other sites. Histologically, the most common subtype was well differentiated liposarcoma (32.5%), followed by myxoid (27.5%), round cell (23.7%), and pleomorphic liposarcoma (16.3%). Forty-eight patients were low-grade liposarcoma (60.0%) and 32 patients were high-grade liposarcoma (40.0%). There were 61 (76.3%) primary liposarcomas and 19 (23.7%) recidivating liposarcomas. Statistical analysis revealed that Eag1 expression is not dependent on age, gender, site, histology, grade, and type in 80 liposarcoma specimens (Table 2).

### 3.3. The Correlation of Liposarcoma Histology with Eag1 Expression

Histological subtype based on morphologic appearance of the tumor is the most important prognostic factor for survival. Previous studies have shown that well differentiated liposarcoma and myxoid have favorable prognosis while poorly differentiated liposarcomas have a poor prognosis [20]. To investigate the correlation between Eag1 expression level and liposarcoma histology and/or clinical outcome, we analyzed Eag1 expression level using the score system (staining intensities of 1+ were considered as low Eag1 expression and 2-3+ were considered as high Eag1 expression); Eag1 expression in different liposarcoma histological subtypes was shown in Figure 2. High Eag1 expression was detected in 23 cases (42.6% of the positive expression cases), while the other 31 cases (57.4%) showed low Eag1 expression. There was a clear difference in Eag1 expression levels between well differentiated liposarcoma (21.1%) and pleomorphic/round cell liposarcoma. Meanwhile the high expression rate of Eag1 in myxoid liposarcoma (40.0%) was lower than in pleomorphic and round cell liposarcoma (66.7% and 63.6%, resp.), but the difference was not statistically significant (Table 3).

### 3.4. Eag1 Blockage Reduces the Proliferation of Liposarcoma Cells

To characterize the oncogenic role of Eag1 in liposarcoma, we first inhibited Eag1 expression by Eag1 shRNA. As shown in Figure 3(a), Eag1 protein expression was effectively suppressed by Ad5-Eag1-shRNA. Next the effect of Eag1 knockdown on cell proliferation was determined by CCK-8 assay. The results revealed that the proliferation of SW-872 and 93T449 cells was inhibited by 39% and 31%, respectively, after Ad5-Eag1-shRNA infection. To confirm the oncogenic role of Eag1, we treated liposarcoma cells with imipramine, a nonspecific blocker of Eag1 activity. The results showed that the proliferation of SW-872 and 93T449 cells was inhibited by 28% and 22%, respectively, after the treatment with 20 *μ*M imipramine (Figure 3(b)). Similar results were obtained from the colony formation experiment (Figure 3(c)). Collectively, these results suggest that Eag1 promotes the proliferation of liposarcoma cells* in vitro*.

### 3.5. Eag1 Silencing Inhibits Liposarcoma Growth* In Vivo*

To investigate the* in vivo* role of Eag1 in liposarcoma, we made a xenograft model of liposarcoma using nude mice and treated the xenografts by intratumor injection of Ad5-Eag1-shRNA, Ad5-Control-shRNA, or saline (Figure 4(a)). The results showed that the tumor volume was significantly smaller in Ad5-Eag1-shRNA injected animals than in saline or Ad5-Control-shRNA injected animals at each evaluating time point (Figure 4(b)). These* in vivo* data confirm our* in vitro* results and suggest the oncogenic role of Eag1 in liposarcoma.

### 3.6. Eag1 Silencing Inhibits Cell Cycle Progression of Liposarcoma Cells

To determine how Eag1 knockdown inhibits liposarcoma growth, we analyzed DNA contents of SW-872 and 93T449 cells by flow cytometry. As shown in Figure 5, Ad5-Eag1-shRNA led to accumulation of cells in the G1 phase (*n* = 3, *P* < 0.01) and reduction of cells in the G2 phase, while it demonstrated no effect on the S phases of the cell cycle in two liposarcoma cell lines. The results suggested that Eag1 is important for the cell cycle of SW-872 and 93T449 cells which are consistent with conclusions reported by others that Eag1 is necessary for progression through the G1 phase and G0/G1 transition of the cell cycle [21].

### 3.7. Eag1 Silencing Reduces p38 MAPK Activity in Liposarcoma Cells

To explore the molecular mechanism underlying the oncogenic role of Eag1 in liposarcoma, we focused on p38 MAPK pathway because Eag1 has been shown to activate p38 MAPK pathway [22], which is frequently activated in a variety of tumors [23]. Western blot analysis showed that the level of phospho-p38 MAPK was lower in Ad5-Eag1-shRNA infected SW-872 and 93T449 cells than in negative control cells (Figure 6). Taken together, these data indicate that Eag1 knockdown may inhibit the activation of p38 MAPK which then promotes growth and cell cycle arrest in liposarcoma cells.

## 4. Discussion

Although surgery and radiation therapy could achieve good results for liposarcoma, it is difficult for complete surgical removal of liposarcoma within the abdomen. Moreover, distant metastasis remains a therapeutic dilemma limiting the survival of liposarcoma patients [24]. Therefore, there is an urgent need to identify novel targets for the diagnosis, prognosis, and therapy of liposarcoma.

Based on histological findings and cytological aberrations, liposarcomas are classified into four subtypes: well differentiated, myxoid, pleomorphic, and round cell. Subtype is the most important determinant of clinical outcome and different subtypes have clearly different effects on survival analysis [25]. Some clinical criteria, such as gender, age, location, histology, and size, can be used to estimate patient outcome [26]. However, a significant variability in predictive value exists among different clinical laboratories and hospitals with regard to the assessment of liposarcoma histological subtype. Recently, the alteration in gene expression is proposed to be crucial to malignant transformation and development of malignant phenotype in liposarcomas [27].

Increasing evidence suggests that Eag1 channel is aberrantly expressed in many types of tumors but negatively expressed in noncancerous matched tissues [10]. Additionally, the inhibition of Eag1 expression or Eag1-mediated currents could suppress tumor cell proliferation [14, 28]. Therefore, Eag1 has emerged as a promising target for cancer detection and therapy [15].

In the present study we examined the expression of Eag1 in liposarcoma of patients because of its restricted distribution in normal tissue and its more ubiquitous distribution in cancer cells and its oncogenic properties. We determined Eag1 expression in different adipose tissues diseases from 109 patients by immunohistochemistry and the data provide evidence that Eag1 is expressed in liposarcoma with a higher frequency compared to lipoma, hyperplasia, inflammation, and normal adipose tissues. However, the expression of Eag1 is not correlated with any clinicopathological features of liposarcoma. The high expression rate of Eag1 is lower in well differentiated liposarcoma specimens than in pleomorphic and round cell liposarcoma, while round cell and pleomorphic liposarcomas have definitely poorer prognosis than well differentiated liposarcomas. Probably due to sample size limitation, the high expression rate of Eag1 in myxoid, round cell, and pleomorphic liposarcomas has no significant difference. Taken together, our data partly indicate an association between Eag1 expression and poor prognosis of liposarcoma patients. However, further studies with long outcome and larger number of patients are needed to clarify the potential of Eag1 as a prognostic marker in liposarcoma.

To establish a useful model for further studies, we tested the role of Eag1 in two well-established liposarcoma cell lines (SW-872 and 93T449). We observed a significant reduction of proliferation and colony formation in two cell lines after treatment with 20 *μ*M imipramine, which is in good agreement with previous studies [16, 29, 30]. However, imipramine could pass the blood-brain barrier and have effects on intracranial Eag1 [31]. Compared with imipramine, siRNA is a more specific tool to investigate the role of Eag1 in cancer progression. siRNA mediated knockdown of Eag1 results in reduced proliferation of tumor cells without observable nonspecific responses [12]. In our study, Eag1-shRNA could effectively inhibit the proliferation and growth of liposarcoma cells* in vitro* and* in vivo*. Proliferation inhibition can be a result of cell cycle arrest, so next flow cytometry was used to detect the effects of Eag1-shRNA on cell cycle. It was found that Eag1-shRNA significantly affected the cell cycle, which increased the percentage of cells in G1.

Eag1 overexpression is known to be implicated in tumor progression. However, the intracellular signaling pathways downstream of Eag1 has not been fully characterized. Although Eag1 channel is a transmembrane protein, potassium permeation is not the only feature of its relevance to tumor progression [31]. So Eag1 blockers could reduce proliferation not only by inhibiting permeation, but also by trapping Eag1 in a particular conformation [32]. We chose to focus on p38 MAPK pathway because of its critical roles in the pathogenesis of various cancers, including liposarcoma [33]. It has been proposed recently that perinuclear localization of Eag1 could lead to the activation of MAPK pathway, resulting in increased cell proliferation [15]. Moreover, new functions for p38 MAPK have been elucidated in recent years and one of these functions is the regulation of the cell cycle and checkpoint controls [34]. Interestingly, Several K^+^ channels including Eag1 are often overexpressed in tumor cells and regulate proliferation. They are needed to control specific checkpoints in the cell cycle progression [35]. We demonstrated that Eag1 knockdown inhibits the activation of p38 MAPK which then may induce the growth and cell cycle arrest of liposarcoma cells. Therefore, it is possible that Eag1 overexpression induces the activation of p38 MAPK and promotes tumorigenesis. Collectively, our data demonstrate that Eag1 is overexpressed and plays oncogenic role in liposarcoma. Eag1 may present a potential therapeutic target for liposarcoma. However, further studies are needed to clarify the potential of Eag1 as a prognostic marker in liposarcoma.

## Figures and Tables

**Figure 1:** The expression of Eag1 in different adipose tissues diseases samples. (a) Real-time PCR reveals increased Eag1 expression in liposarcoma. The mRNA expression level is normalized with GAPDH and the value in normal adipose tissues is set as 1 for the calibration. ^∗∗∗^ *P* < 0.001. (b) Eag1 immunostaining in a human brain specimen (positive control, (A)), 67.5% liposarcoma (B), 42.1% lipoma (C), 40.0% hyperplasia of adipose tissues (D), 25.0% panniculitis (E), and no positive Eag1 staining in 9 normal adipose tissues (F) and 3 skeletal muscle tissues (negative control, (G)). Images are captured using an OLYMPUS light microscope equipped with a CCD color camera at a 200x magnification.

**Figure 2:** Immunohistochemical staining of Eag1 in different liposarcoma samples. Examples of high expression levels of Eag1 in myxoid liposarcoma (a), pleomorphic liposarcoma (b), round cell liposarcoma (c), and well differentiated liposarcoma (d). Low expression levels of Eag1 are shown in myxoid liposarcoma (e), pleomorphic liposarcoma (f), round cell liposarcoma (g), and well differentiated liposarcoma (h). Magnification: 40x.

**Figure 3:** Eag1 blockage inhibits the proliferation and tumorigenicity of liposarcoma cells. (a) Western blot analysis of Eag1 protein levels in liposarcoma cells treated with Eag1 shRNA. Densitometric analysis of the bolts with GAPDH as loading control. The results are expressed as mean ± SD (*n* = 3). (b) The proliferation of liposarcoma cells is determined by CCK-8 assay after treatment with imipramine or Eag1 shRNA. The proliferation of liposarcoma cells is significantly reduced after treatment with imipramine or Eag1 shRNA. Data are presented as mean ± SD (*n* = 6). (c) The tumorigenicity of liposarcoma cells is determined by colony formation assay. The tumorigenicity of liposarcoma cells is significantly reduced after treatment with 20 *μ*M imipramine or Eag1 shRNA. Data are presented as mean ± SD (*n* = 3). ^∗∗^ *P* < 0.01.

**Figure 4:** Ad5-Eag1-shRNA inhibits liposarcoma growth* in vivo*. (a) Cartoon representation of the experiment with liposarcoma xenograft tumors and Ad5-Eag1-shRNA treatment. Xenograft tumors are established by subcutaneous injection of 1 × 10^5^ liposarcoma cells. After two weeks, the tumors grow to visible size. Ad5-Eag1-shRNA treatment is given by intratumor injection every third day (blue arrows). Mice in the control group are injected with saline or Ad5-Control-shRNA. (b) The length and width of tumors are measured every third day after inoculation and the volume of tumor is calculated. After 15 days, the tumor volume growth curve is drafted. ^∗∗^ *P* < 0.01 versus saline or Ad5-Control-shRNA group.

**Figure 5:** The effects of Eag1 silencing on the progression of cell cycle. Cells were infected with shRNA for 48 h. (a) Eag1 silence induced a significant increase in SW-872 cells arrested in the G1 phase (*P* < 0.01, *n* = 3) and a decrease in cells arrested in the G2 phase, while it demonstrated no effect on the S phases of the cell cycle. Representative images of negative control, Ad5-Control-shRNA, and Ad5-Eag1-shRNA group. (b) Similar results were obtained from 93T449 cells.

**Figure 6:** Eag1 regulates p38 MAPK activity in liposarcoma cells. Cells were infected with shRNA for 48 h. (a) Western blot analysis of phosphorylated p38 MAPK level in Ad5-Eag1-shRNA group and negative control group. (b) Densitometric analysis of the blots with GAPDH as loading control. Data are expressed as mean ± SD (*n* = 3). ^∗∗∗^ *P* < 0.001.

**Table 1:** The expression of Eag1 in different adipose tissues diseases.

Histology	Number of tumors (%)	Eag1 expression (%)	*χ* ^2^ value	*P*
Liposarcoma	80 (61.1%)	54 (67.5%)		
Lipoma	19 (14.5%)	8 (42.1%)	4.23	0.04
Hyperplasia of adipose tissues	15 (11.5%)	6 (40.0%)	4.11	0.043
Panniculitis (inflammation)	8 (6.1%)	2 (25.0%)	5.68	0.017
Normal adipose tissues	9 (6.9%)	0 (0.0%)	15.448	<0.001

Total	131	70 (53.4%)		

**Table 2:** Clinical Parameters of liposarcoma specimens and Eag1 expression.

Clinical parameters of samples	Number of tumors (%)	Eag1 expression (%)	*χ* ^2^ value	*P*
Sex			0.382	0.536
Male	33 (41.2%)	21 (63.6%)		
Female	47 (58.8%)	33 (70.2%)		
Age (year)			0.166	0.983
≤30	4 (5.0%)	3 (75.0%)		
30–39	25 (31.3%)	17 (68.0%)		
40–60	34 (42.5%)	23 (67.6%)		
>60	17 (21.2%)	11 (64.7%)		
Site			0.735	0.865
Limbs	21 (26.2%)	13 (61.9%)		
Trunk	23 (28.8%)	15 (65.2%)		
Abdominal cavity	21 (26.2%)	15 (71.4%)		
Other	15 (18.8%)	11 (73.3%)		
Histology			1.19	0.755
Well differentiated	26 (32.5%)	19 (73.1%)		
Myxoid	22 (27.5%)	15 (68.2%)		
Pleomorphic	13 (16.3%)	9 (69.2%)		
Round cell	19 (23.7%)	11 (57.9%)		
Grade			1.605	0.205
Low-grade	48 (60.0%)	35 (72.9%)		
High-grade	32 (40.0%)	19 (59.4%)		
Type			0.214	0.644
Primary	61 (76.3%)	42 (68.9%)		
Recurrence	19 (23.7%)	12 (63.2%)		

Total	80	54 (67.5%)		

**Table 3:** Tumour histology and dichotomised Eag1 expression.

	Low Eag1 expression (%)	High Eag1 expression (%)	*χ* ^2^ value	*P*
Histology				
Well differentiated	15 (78.9%)	4 (21.1%)		
Myxoid	9 (60.0%)	6 (40.0%)	1.449	0.229
Pleomorphic	3 (33.3%)	6 (66.7%)	5.535	0.035
Round cell	4 (36.3%)	7 (63.6%)	5.44	0.047

Total	31 (57.4%)	23 (42.6%)		
